This article has been retracted.

# Identification of a Novel Jasmonate-Responsive Element in the *AtJMT* Promoter and Its Binding Protein for *AtJMT* Repression

**DOI:** 10.1371/journal.pone.0055482

**Published:** 2013-02-05

**Authors:** Jun Sung Seo, Yeon Jong Koo, Choonkyun Jung, Song Yion Yeu, Jong Tae Song, Ju-Kon Kim, Yeonhee Choi, Jong Seob Lee, Yang Do Choi

**Affiliations:** 1 Department of Agricultural Biotechnology, Seoul National University, Seoul, Korea; 2 School of Applied Biosciences, Kyungpook National University, Daegu, Korea; 3 School of Biotechnology and Environmental Engineering, Myongji University, Yongin, Korea; 4 School of Biological Sciences, Seoul National University, Seoul, Korea; Ohio State University, United States of America

## Abstract

Jasmonates (JAs) are important regulators of plant biotic and abiotic stress responses and development. *AtJMT* in *Arabidopsis thaliana* and *BcNTR1* in *Brassica campestris* encode jasmonic acid carboxyl methyltransferases, which catalyze methyl jasmonate (MeJA) biosynthesis and are involved in JA signaling. Their expression is induced by MeJA application. To understand its regulatory mechanism, here we define a novel JA-responsive *cis*-element (JARE), G(C)TCCTGA, in the *AtJMT* and *BcNTR1* promoters, by promoter deletion analysis and Yeast 1-Hybrid (Y1H) assays; the JARE is distinct from other JA-responsive *cis*-elements previously reported. We also used Y1H screening to identify a *trans*-acting factor, AtBBD1, which binds to the JARE and interacts with AtJAZ1 and AtJAZ4. Knockout and overexpression analyses showed that AtBBD1 and its close homologue AtBBD2 are functionally redundant and act as negative regulators of *AtJMT* expression. However, AtBBD1 positively regulated the JA-responsive expression of *JR2*. Chromatin immunoprecipitation from knockout and overexpression plants revealed that repression of *AtJMT* is associated with reduced histone acetylation in the promoter region containing the JARE. These results show that AtBBD1 interacts with JAZ proteins, binds to the JARE and represses *AtJMT* expression.

## Introduction

Jasmonic acid and its derivatives, collectively referred to as jasmonates (JAs), act as important regulators in plant biotic and abiotic stress responses [1], [2], [3]. JA also plays important roles in physiological and developmental processes, including root growth, senescence, trichome formation, cell cycle progression, and flower development [4], [5].

The molecular mechanisms by which JA regulates gene expression were illuminated by the discovery of jasmonate ZIM-domain proteins (JAZs) and the finding that the SCF^COI1^ complex-mediated 26S proteasome degrades JAZs [6], [7]. In the absence of JA, JAZ proteins bind to transcription factors (TFs) and prevent their activity by recruiting the general co-repressor TOPLESS (TPL), through interaction with the adaptor protein Novel Interactor of JAZ (NINJA) [8], or by directly recruiting histone-modifying proteins, such as histone deacetylases (HDACs) [9], [10]. In the presence of the signal, JA is converted into jasmonoyl-isoleucine (JA-Ile) by JAR1 in *Arabidopsis* [11], [12]. JA-Ile then promotes the interaction between JAZ proteins and the F-box protein Coronatine insensitive1 (COI1), in the SCF complex, resulting in proteolytic degradation of JAZ proteins by the 26S proteasome [6], [7]. Degradation of JAZ proteins liberates TFs from NINJA, TPL or HDACs, and initiates transcriptional reprogramming in response to JA [13], [14].

Recent reports on JA-responsive TFs have further improved our understanding of JA-responsive regulatory mechanisms. AtMYC2, a bHLH TF, is a primary target in the JA signaling pathway and interacts with some members of the AtJAZ family to regulate various JA-responsive target genes [15], [16], [17]. Other TFs also have been shown to interact with specific JAZ proteins [18], [19], [20]. It has been speculated that the specific interactions between TFs and JAZs could be largely responsible for the specificity and diversity of JA responses to different stimuli [21], [22].

These TFs bind to specific promoter elements of downstream genes and propagate JA signaling. One well-defined JA-responsive element, which is bound by MYC2, is the G-box (CACGTG) or G-box like motif (core ACGT) [17]. The G-box has been found in the promoters of many JA-responsive genes, such as *VSP1* in *Arabidopsis* [23], *PIN2* in potato [24], *VSPB* in soybean [25], and *ORCA3* in *Catharanthus* [26]. Another JA-responsive element is the GCC-motif in *PDF1.2* in *Arabidopsis* [27], *PMT* in tobacco [28] and *STR* in *Catharanthus* [29]. Other JA-responsive sequence motifs have also been reported [30], [31]. Transcriptome shifts of gene clusters responding to hormonal signals closely corresponded with the set of *cis*-elements in the genes’ promoters [32]. Some elements are involved in signal transduction in response to a specific hormone; others respond to two or more hormonal signals [33]. Therefore JA-responsive *cis*-elements are key to understanding both JA-specific signal transduction and inter-hormonal cross-talk.

Histone acetyltransferases (HATs) and histone deacetylases (HDACs) play key roles in regulating gene expression through histone modification. The addition of acetyl groups to conserved lysine residues neutralizes the positive charge of histone tails and decreases their affinity for DNA [34], [35]. Hypoacetylation mediated by HDACs has the opposite effect on chromatin, enabling the histones to bind more tightly to the negatively-charged DNA, and is associated with the repression of gene expression [36], [37]. HATs and HDACs interact with co-activator and co-repressor complexes, respectively, to regulate expression of target genes [38], [39]. There are reports that transcription levels of some JA-responsive genes are altered in *Arabidopsis HDAC6* or *HDAC19* knockout mutants and overexpression plants [40], [41].

One key aspect of JA signaling is feedback regulation of JA synthesis. In *Arabidopsis*, the expression of *AtJMT*, which encodes a jasmonic acid carboxyl methyltransferase responsible for MeJA formation, is developmentally regulated and induced upon wounding or JA application [42]. *BcNTR1* encodes the orthologous JA carboxyl methyltransferase in *Brassica campestris* [43] and its expression pattern is similar to the pattern of *AtJMT* expression. In this study, we identified a novel JA-responsive *cis*-element (JARE) in the *AtJMT* and *BcNTR1* promoters and isolated a *trans*-acting factor, AtBBD1, which binds to the JARE and interacts with AtJAZ1 and AtJAZ4. We also showed that AtBBD1 regulates transcription of *AtJMT* and another JA-regulated gene.

## Materials and Methods

### Plant Materials and Treatments

*Arabidopsis thaliana* ecotype Columbia (Col-0) was used as the wild type for all experiments. The *Brassica campestris* variety and source were described in Song et al. (2000) [44]. Plants were grown on soil or one-half-strength Murashige and Skoog agar medium (Duchefa) in a growth chamber maintained at 22°C and 60% relative humidity under long-day conditions (16-h-light/8-h-dark cycle). *Arabidopsis* was transformed with *Agrobacterium tumefaciens* (strain C58C1) using the ﬂoral dip method [45]. A construct list of transgenic plants used in this study is provided in Supplemental Table 1 online. Transformed lines (T1 generation) were selected on MS plates containing kanamycin (30 µg/ml) or hygromycin (20 µg/ml). At least 40 independent T1 plants per genotype were tested for *GUS* expression in response to JA. We identified homozygous lines by testing T3 progeny for resistance to antibiotics. The basal level and MeJA responsive induction of reporter gene were variable among transformants. A line showing medium level of expression was selected from each construct by RT-PCR analysis. Several lines showing extremely high or low level of basal expression were excluded. For chemical treatment, solutions of 100 µM MeJA (Aldrich), 100 µM (±)-JA (Duchefa), 100 µM (±)-ABA (Duchefa), 50 µM SA (Sigma), or 5 mM ethephon were applied to soil-grown 4-week-old plants by spraying.

### Y1H and Y2H Assays

The yeast one-hybrid screening was performed using MATCHMAKER One-Hybrid Library Construction and Screening Kit (Clontech). To isolate JARE-binding proteins_,_ a cDNA library was prepared by RT-PCR from MeJA-treated seedlings of *Arabidopsis* Col-0 into pGADT7-Rec2. Bait DNA (−3518 to −3390 bp) containing JARE was cloned into the pHIS2 reporter vector. Positive clones were identified by nucleotide sequencing with AD sequencing primers. To identify the AtBBD1 binding sequence, various promoter fragments were cloned into the pHIS2 vector. The full length CDS or specific domains of AtBBD1 were cloned into pGADT7-Rec2.

Y2H assays were carried out using the MATCHMAKER Two-Hybrid System (Clontech). Full-length cDNAs for 12 *AtJAZ* genes were amplified by RT-PCR from 14-day-old seedlings of *Arabidopsis* Col-0 (Table S1). Each gene was cloned into the Y2H prey vector, pGADT7, to get the prey gene construct. The full-length coding region of *AtBBD1* was amplified by RT-PCR and cloned into the Y2H bait vector, pGBKT7. All constructs used in Y1H and Y2H are shown in Table S1.

### Electrophoretic Mobility Shift Assay

Full length CDS or DNA binding domain (a.a. residue 257 to 325) of AtBBD1 were fused in frame with the maltose-binding protein (MBP) at the C-terminus and expressed in *Escherichia coli.* A soluble crude extract of recombinant protein was used for EMSA. DNA fragments labeled with [γ-^32^P]dCTP were incubated with MBP-AtBBD1 or MBP-AtBBD1DB in the binding buffer [20 mM HEPES, pH 7.9, 50 mM KCl, 0.5 mM DTT, 1 mM EDTA, 10% glycerol, 5 mM MgCl2, 0.01% Triton X-100, and 100 ng poly(dI-dC)] for 1 hour. For competition analysis, unlabeled DNA fragments were included in the binding reactions as competitors in 10-fold molar excess relative to the labeled probes in each step. The reaction mixture was analyzed by 10% polyacrylamide gel electrophoresis and the wet gel was exposed and detected by BAS reader (BAS-2010, Fujifilm).

### Northern Blot and RT-PCR Analysis

Northern blot analysis and RT-PCR were carried out as described by Seo et al. (2011) [46]. Primer pairs used to amplify cDNA probes are listed in Table S1. For RT-PCR analysis, first-strand cDNA was synthesized from 2 ug of total RNA with oligo(dT)_15_ using Superscript III reverse transcriptase (Invitrogen) according to the manufacturer’s instructions. PCR was performed using sequence-specific primers described in Table S1 with 24 cycles, which was optimized to be within the linear range of amplification.

### *In Vitro* Pull-down Assay

*In vitro* pull-down assays were carried out according to the procedure of Seo et al. (2011) [46]. The full length CDS of *AtJAZ1* was fused in frame with the maltose-binding protein (MBP) at the C-terminus in pMAL-c2E vector, expressed in *Escherichia coli* and purified using amylose resin. Pulled-down mixtures were separated by SDS–PAGE, transferred to nitrocellulose membrane (Whatman), and detected using anti-c-myc antibody (Santa Cruz Biotechnology).

### Agroinfiltration and Transient Protein Expression

Agroinfiltration for transient protein expression in tobacco leaves was performed according to the method described by Voinnet et al. [47], with minor modifications. Briefly, *Agrobacterium tumefaciens* strains C58C1 carrying either the 6xMYC-BBD1 or 3xHA-AtJAZ1 construct under the control of the 35S promoter were grown at 28°C in Luria-Bertani medium and resuspended in infiltration media. For cotransfections, *Agrobacterium* cultures carrying each construct were mixed in equal proportion. Leaves of 4-week-old *Nicotiana benthamiana* plants were infiltrated with a needleless syringe carrying bacterial cultures through the abaxial air spaces.

### Chromatin Immunoprecipitation

ChIP-PCR was carried out as described by Saleh et al. (2008) [48]. Anti-acetylated H4K12 and anti-acetylated H3K14 antibodies were purchased from Upstate. After immobilization using protein A agarose (Pierce), bound DNA was eluted and amplified by primers corresponding to sequences neighboring the AtBBD1 binding sites in the promoter of *AtJMT*. PCR products were separated on ethidium bromide-stained agarose gel or real-time PCR was used to quantify the amplification. For real-time PCR, amplification of *P_JMT_* (near the JARE) was normalized to that of Actin [49]. Chromatin precipitated without antibody was used as a negative control, and the chromatin before precipitation was used as the input control. ChIP assays were independently repeated twice with the same result. Real-time qRT-PCR was performed using a LightCycler 480 II machine (Roche Diagnostics) with a SYBR Premix EX Taq Kit (TaKaRa). Primers used for qRT-PCR are listed in Table S1. Each qRT-PCR was independently repeated three times with the same expression pattern.

## Results

### The Promoter Regions of *BcNTR1* and *AtJMT* Contain a JA-responsive Element

*AtJMT* and *BcNTR1* are orthologues, which are both induced by MeJA treatment [42], [43], [44]. To understand the regulatory mechanism of *BcNTR1* and *AtJMT* JA-responsive expression, we first defined the promoter regions that mediate induction by JA. Promoter regions 4.4 kb upstream of *BcNTR1* and 4.5 kb upstream of *AtJMT,* respectively, were combined with the *GUS* coding sequence and transformed into *Arabidopsis*. Transcription of *GUS* was induced within 1 hour after MeJA treatment in both sets of transgenic plants (Figure 1), showing that these promoter regions could recapitulate JA-responsive induction. These results indicate that both fragments contain putative JA-responsive *cis*-acting elements (JARE). Also, these results showed that the *BcNTR1* promoter works in *Arabidopsis* although it originated from *Brassica.*

**Figure 1:** *AtJMT* and *BcNTR1* promoters contain JA-responsive transcriptional regulatory elements. Northern blot analysis of the recombinant *GUS* gene after MeJA treatment of transgenic *Arabidopsis*. *BcNTR1* (4.4 kb length, A) and *AtJMT* (4.5 kb length, B) promoters fused to the *GUS* gene are shown. Nucleotide sequence of the promoter is numbered from translation initiation site.

### Identification of a JARE in the *AtJMT* Promoter

We next used promoter-deletion analysis to locate the JARE(s) present in the *AtJMT* promoter. A series of 5′-deleted promoters was fused to the *GUS* coding region and transformed into *Arabidopsis*. Each construct contains from 4.5 kb to 500 bp of the promoter region (Figure 2A). *GUS* expression in response to MeJA treatment was examined by RT-PCR. When MeJA was applied, transgenic plants containing promoter fragments longer than 2.0 kb (JP4.5∼JP2.5) showed *GUS* induction within 1 hour; however, those containing promoter fragments shorter than 2.0 kb (JP2.0∼JP0.5) did not show *GUS* induction (Figure 2A). These results indicate that a putative JARE is located in the 500 bp region between position −2500 and −2000 bp in the *AtJMT* promoter.

**Figure 2:** Localization of the JA-responsive *cis*-element (JARE) in the *AtJMT* promoter. (A) A series of 5’ deleted promoters (closed bar) was cloned upstream of *GUS* coding region (open bar) and transformed into *Arabidopsis*. RT-PCR analysis of each transgenic plant was carried out after 1 hour of MeJA treatment. The JARE is located in the region between −2500 and −2000. (B) Additional promoter deletion constructs between −2500 and −2000 are shown and their *GUS* gene expression in response to MeJA treatment is shown. The putative JARE is located in the region between −2294 and −2280 (gray bar). The positions of the G-boxes are shown at −2529, −2406 and −2342 (▾).

To narrow down the position of the JARE, we generated additional 5′ deletion constructs subdividing the −2,400 to −2,000 bp region of the *AtJMT* promoter. As before, promoter regions were fused to *GUS* and transformed into *Arabidopsis*. When *GUS* mRNA levels were analyzed by RT-PCR after MeJA treatment, constructs containing 2,400 and 2,294 bp of the *AtJMT* promoter were responsive to MeJA, but constructs containing regions shorter than 2,294 bp were not responsive to MeJA (Figure 2B). Therefore, the putative JARE is located in the 15 bp region between the positions −2,294 and −2,280 bp of the *AtJMT* promoter.

### Identification of a JARE in the *BcNTR1* Promoter

In parallel, a series of *BcNTR1* promoter deletion constructs was made and transformed into *Arabidopsis* to identify the JARE in *BcNTR1_._ GUS* mRNA levels were examined by RT-PCR and were induced rapidly, within 1 hour after MeJA treatment, in NP4.0 but not in NP3.0 and NP2.0 lines. Another construct, NPfr1, containing a 3,807 bp fragment of the *BcNTR1* promoter with a deletion between −3,108 and −446, showed a similar response to NP4.0 (Figure 3A). These results showed that the region between −3,807 and −3,256 in the *BcNTR1* promoter also contains a JARE. To test this hypothesis, an additional deletion construct, NP4-A, was made, in which the −3,518 to −3,480 region was deleted. When transgenic *Arabidopsis* plants containing the NP4-A construct were treated with MeJA, these lines showed no induction of *GUS* (Figure 3B). These results show that the JARE is localized in the 39 bp region, between −3,518 and −3,480 bp of the *BcNTR1* promoter.

**Figure 3:** Localization of JARE in the *BcNTR1* promoter. (A) Structures of promoter deletion constructs of *BcNTR1* for JA response tests (left) and RT-PCR analysis of transgenic *Arabidopsis* after MeJA treatment (right). The JARE is located in the region between −3807 and −3256. (B) The *BcNTR1* promoter has a region A (−3518 to −3480) of sequence identity with the *AtJMT* promoter in NPfr1. In the NP4-A construct, the A region was deleted from NP4.0. *GUS* was analyzed by RT-PCR in transgenic plants after MeJA treatment. JARE resides in the A region, −3518 to −3480. (C) Sequence alignment between putative JARE-containing regions in JP2294 of Fig. 2B and A region in NPfr1. Sequence elements (putative JARE) that are identical between JP2294 and NP4-A_._ are shown in bold.

Sequence alignment between the JARE-containing regions of the *AtJMT* promoter (15 bp) and the *BcNTR1* promoter (39 bp) showed a highly conserved sequence motif, TCCTGA (Figure 3C). We hypothesized that this conserved sequence element is a putative JARE (TCCTGA) that could play a critical role in the JA responsiveness of *AtJMT* and *BcNTR1* expression.

### A Multimerized JARE-containing Construct Responds to MeJA

To show regulation of JA responses by the JARE, we next made a construct containing multimers of the JARE-containing promoter region linked to a minimal promoter and tested whether it could mediate JA-responsive induction of transcription. A region containing the putative JARE, between −2305 and −2278 of the *AtJMT* promoter, was duplicated 4 times and fused with the TATA-box sequence (−46 to +8) of the CaMV 35S promoter and a GUS coding sequence. Also a mutant version, in which the core 6 nucleotides, TCCTGA, were mutated to TTTTTT, was constructed in the same manner to determine the role of this core element in response to JA (Figure 4A). All the constructs were transformed into *Arabidopsis* (Col-0) and transgenic lines were treated with MeJA. Histochemical staining of transgenic plants showed that JA-responsive GUS activity was present only in 4xJARE:GUS lines, but not in 4xmJARE:GUS lines (Figure 4B). RT-PCR analysis also showed that GUS transcript was induced within 1 hour in 4xJARE:GUS lines (#17 and # 25) in response to MeJA, but was not induced in 4xmJARE lines (#12 and #31) (Figure 4C). Taking these data together, we concluded that the conserved 6-nucleotide element (TCCTGA) in the *AtJMT* and *BcNTR1* promoters is indeed a JARE.

**Figure 4:** JARE-containing transgenic plants show MeJA response. (A) Schematic representation of multimerized JARE- containing construct (4xJARE:GUS), and its mutant version (4xmJARE:GUS). The DNA fragment from the *AtJMT* promoter (−2305 to −2278) containing the JARE was repeated 4 times and recombined to the GUS reporter containing a minimal promoter (TATA) from CaMV 35S. JARE(TCCTGA) and its mutant version are shown in bold. (B) Histochemical staining of 4xJARE:GUS (#17) and 4xmJARE:GUS (#12) transgenic plants with (+) or without (−) MeJA treatment for 4h. (C) RT-PCR analysis of *GUS* in each transgenic line was carried out after MeJA treatment.

### Identification of a JARE-binding Protein

We next carried out yeast one-hybrid (Y1H) screening to isolate protein factors that bind to the JARE. A segment (−3,518 to −3,390) of the *BcNTR1* promoter containing the JARE was employed as bait in the reporter construct. The yeast cells were co-transformed with activator constructs incorporating cDNA libraries prepared from MeJA treated *Arabidopsis*. Clones were sequenced from positive colonies and sequence analysis showed that multiple positive clones corresponded to *AtBBD1* (Figure S1). *AtBBD1* is an *Arabidopsis* homologue of the *Oryza minuta bifunctional nuclease in basal defense response* (*OmBBD1*), which acts in abscisic-acid (ABA)-dependent callose deposition [50]. The *Arabidopsis thaliana* genome also contains an *AtBBD1* homologue, *AtBBD2,* with 81% amino acid sequence identity to *AtBBD1* (Figure S2C).

To determine whether AtBBD1 binds to the putative JARE core sequence of GTCCTGA in the *BcNTR1* promoter fragment, or to another *cis*-element, the bait region (−3518 to −3390) of the *BcNTR1* promoter was divided into three segments; a (−3518 to −3471), b (−3471 to −3430) and c (−3430 to −3390) (Figure 5A). Each segment was tested for interaction with AtBBD1 by Y1H assay. AtBBD1 was fused with the activation domain of GAL4 (AD) in the activator construct. These assays showed that AtBBD1 bound only to the segment (−3518 to −3471) that contains the GTCCTGA core sequence.

**Figure 5:** Identification of sequence element in the *BcNTR1* promoter region to which AtBBD1 binds. (A) Structures of reporter and activator genes used in Y1H assays. The promoter region of *BcNTR1*, −3518 to −3390, was divided into 3 segments and each segment was used as bait for Y1H assays. The control does not contain any of those segments. AtBBD1 was fused with the GAL4 activating domain (AD) as an activator. The position of the putative JARE is shown (▾). (B) The segment a was divided further into 8 subsegments (6 nt each) and each subsegment, a1 to a8, was mutated into 6 adenines. Each mutant segment was tested as bait in Y1H assays. (C) Subsegments a6 and a7 to which AtBBD1 bound, were dissected further by mutation in overlapping frames. In each mutant, 6 nucleotides were mutated into 6 adenines. Each mutant subsegment, M0–M5, was tested by Y1H assays. The sequence motif to which AtBBD1 binds is shown in bold. (D) Mutation analysis of the AtBBD1 binding element. Mutant series (CM1 to CMR) of JARE was created by changing a single nucleotide from purine to pyrimidine, or *vice versa*, in the fragment −2305 to −2278 as shown in Fig. 4A as a bait and Y1H assays were carried out with AD-AtBBD1. CMR is a JARE in reverse orientation_._

To further narrow down the binding sequences within this segment (−3518 to −3471), a series of mutated bait segments (a1 to a8) was designed by changing 6 nucleotides of each subsegment into 6 adenines (Figure 5B) and testing by Y1H whether these changes affected AtBBD1 binding. AtBBD1 did not bind mutant segments a6 and a7 in yeast; therefore, those 12 nucleotides include sequences necessary for AtBBD1 binding (Figure 5C). Another series of six overlapping mutant constructs, M0–M5, in which 6 nucleotides were mutated into 6 adenines, revealed that the nucleotide element, GTCCTGA, is necessary for AtBBD1 interaction (Figure 5C).

Additional point mutation experiments showed that adenine and thymine in the first nucleotide eliminated AtBBD1 binding (Figure 5D). However, cytosine was acceptable as in P*_JMT_* (see Figure 6). The 7^th^ adenine, which was not tested in the M0–M5 constructs above, was also necessary. The orientation of the heptameric element was also important in the Y1H assay, as the CMR construct, which has the JARE sequence in reverse orientation, did not show AtBBD1 binding in yeast (Figure 5D). In conclusion, the heptameric nucleotide element, G(C)TCCTGA, is critical for AtBBD1 to interact with these DNA sequences (Figure 5D). This result is consistent with the promoter deletion experiments and the multimerized JARE analysis (Figure 4).

**Figure 6:** AtBBD1 and AtBBD2 bind to promoter sequences containing the JARE. Promoter segments, P*_NTR1,_* (−3497 to −3470 of *BcNTR1* promoter) or P*_JMT_* (−2305 to −2278 of *AtJMT* promoter) were used as bait in Y1H assays. A mutated segment, P*_G-box_*, which contains G-box sequence in P*_NTR1_* was used as a bait and an empty vector (pHIS2) was used as a control. AtBBD1 and AtBBD2 were fused with AD. G-box is AtMYC2 binding element (CACGTG) (Boter et al., 2004).

### JARE is Distinct from the G-box

To test the specificity of AtBBD1 binding, Y1H assays were carried out with promoter segments containing different JA-responsive *cis*-elements, including the G-box, placed into the same sequence context as the JARE. For JARE-containing constructs, P*_NTR1_* (−3497 to −3470 of the *BcNTR1* promoter) or P*_JMT_* (−2305 to −2278 of the *AtJMT* promoter), which contain the JARE, were used as bait in the Y1H assay. For the G-box, P*_G-box_* is a mutant version of P*_NTR1_* in which the JARE was replaced with a G-box. The G-box is a typical JA-responsive element and is bound by AtMYC2 [15]. Y1H results showed that AtBBD1 interacted with P*_JMT_* and P*_NTR1_* but did not interact with P*_G-box_* (Figure 6). Therefore, the JARE ((G/C)TCCTGA) of P*_NTR1_* and P*_JMT_*, is a distinct *cis*-element in the *AtJMT* and *BcNTR1* promoters for JA-responsive gene expression. AtBBD1 could regulate expression of *BcNTR1* and *AtJMT* in response to JA through binding to the JARE. AtBBD2, a homologue of AtBBD1, also bound to the same DNA sequences as JARE in Y1H assays (Figure 6).

### The C-terminal Region of AtBBD1 has DNA Binding Activity

Sequence analysis of the AtBBD1 protein family had previously shown that the AtBBD1 proteins contain several conserved domains, including a highly conserved region (HCR), a domain of unknown function 151 (DUF151), and a UV responsive (UVR) domain at the C-terminus [50]. However, this analysis did not identify a known DNA-binding motif; therefore, we tested whether different domains of AtBBD1 had DNA-binding activity. We made five truncated protein constructs (BBD1A-E) each containing one or two domains of AtBBD1 and fused these with AD for Y1H assays to determine their DNA binding activity (Figure 7A). Each construct was co-transformed into yeast with a bait DNA sequence (P*_NTR1_*) that is known to interact with full-length AtBBD1. Constructs BBD1B (116–325) and BBD1E (257–325), which both contain the C-terminal predicted UVR domain, showed DNA binding activity in yeast, but the other constructs showed no DNA binding activity (Figure 7A). This result suggests that the AtBBD1 DNA binding domain resides in the C-terminal region.

**Figure 7:** The DNA binding domain of AtBBD1 resides in the C-terminal region. (A) A schematic representation of truncation mutants of AtBBD1. Numbers indicates amino acid residues, and putative domains are represented (HCR, Highly Conserved Region; DUF151, Domain Unknown Function 151; UVR, putative UV-Response domain) [50]. Each truncated protein was fused with AD as shown in Fig. 5A. P*_NTR1_* (Figure 6) was used as a bait DNA sequence (bottom). (B) Electrophoretic mobility shift assays were carried out using fusion protein (MBP-BBD1) and a 70 bp fragment containing JARE was used as a probe.

To confirm the DNA binding activity of BBD1E (257–325) by electrophoretic mobility shift assays (EMSA), we made a construct, MBP-BBD1E, which fused amino acids 257–325 with Maltose Binding Protein (MBP) and expressed this fusion protein in *E. coli*. Crude extracts containing MBP-BBD1E bound to the 70 bp DNA fragment containing the JARE of the *BcNTR1* promoter. Competition assays with unlabeled probe showed the specificity of binding (Figure 7B). These results show that amino acid residues from 257 to 325 at the C-terminus are involved in DNA binding by AtBBD1.

### AtBBD1 Interacts with the ZIM/TIFY Domain of AtJAZ1 through its HCR Domain

Because JAZ proteins interact with various transcription factors involved in JA-responsive gene expression, we used yeast-two-hybrid (Y2H) assays to test whether AtBBD1 interacts with *Arabidopsis* JAZ proteins. Full-length AtBBD1 was fused to the GAL4 DNA binding domain (BD) and the full-length protein for each of of 12 AtJAZs was fused to the AD. AtBBD1 showed strong interactions with AtJAZ1 and AtJAZ4 in Y2H assays (Figure 8A).

**Figure 8:** AtBBD1 interacts with AtJAZ proteins. (A) Y2H assay between AtBBD1 and each of 12 AtJAZs. Full length CDS of AtBBD1 was fused to GAL4 DNA binding domain (BD) and each full length CDSs of 12 AtJAZs was fused to AD. (B) The pull-down assay between AtBBD1 and AtJAZ1. *35S:6xmyc-AtBBD1* plant extract (input) was incubated with amylose resin bound recombinant MBP-AtJAZ1 protein. Pulled-down protein complex was detected by immunoblotting using anti-MYC antibody (left). MBP protein was used as a pull-down control. The panel on the right shows input recombinant MBP and MBP-AtJAZ1 proteins in the pull-down assay. (C) Immunodetection of the AtBBD1 and AtJAZ1 complex *in vivo.* 35S:6xMYC-AtBBD1 and 35S:3xHA-AtJAZ1 constructs were transiently coexpressed in tobacco leaves by agroinfiltration. The expressed proteins were immunoprecipitated (IP) using anti-HA antibody (+/+) and immunoblotting was carried out with anti-myc antibody. Left lane (−/−) is control leaf extract that was not agroinfiltrated. MYC-AtBBD1 and HA-AtJAZ1 proteins were detected in input coexpressed leaf extracts by each antibody (right). (D) Each truncated AtBBD1 protein was fused to AD as a prey for Y2H assay with AtJAZ1. AtJAZ1 was fused to BD as bait. Numbers indicates amino acid residues, and putative domains were represented. (E) Each truncated AtJAZ1 protein was fused to AD as a prey for Y2H assay with AtBBD1 protein. AtBBD1 was fused to BD as bait.

To confirm the results of the Y2H assay, *in vitro* pull-down assays were carried out. Recombinant MBP-AtJAZ1 bound to amylose resin was incubated with plant extracts prepared from a 35S::6xMYC-AtBBD1 transgenic plant and pulled-down proteins were analyzed by Western blotting with anti-MYC antibody. Recombinant 6xMYC-AtBBD1 was pulled down by recombinant MBP-AtJAZ1 (Figure 8B).

To confirm the interaction between AtBBD1 and AtJAZ1 *in vivo*, 35S:6xMYC-AtBBD1 and 35S:3xHA-AtJAZ1 constructs were transiently coexpressed in tobacco leaves by agroinfiltration. Leaf extract was immunoprecipitated with anti-HA antibody and then immunoblotted with anti-MYC antibody (Figure 8C). These results showed that AtBBD1 directly interacts with AtJAZ1.

To identify the domain of AtBBD1 that mediates interaction with AtJAZs, truncated AtBBD1 proteins were fused with the AD and full length AtJAZ1 was fused with BD for Y2H assays. Y2H results showed that BBD1A (1–116), and H (81–116) interacted with AtJAZ1 in yeast, indicating that the HCR domain between amino acid residues 81 and 116 of AtBBD1 interacts with AtJAZ1 (Figure 8D).

Reciprocally, to identify the domain of AtJAZ1 that mediates interaction with AtBBD1, 5 truncated protein constructs containing the ZIM/TIFY or Jas domains of AtJAZ1 were designed for Y2H assays. JAZ1A (1–204) and JAZ1B (100–181) fragments as well as JAZ1F (full length JAZ1) interact with AtBBD1. These results indicate that the amino acid sequence from 100 to 181 of AtJAZ1, which contains the ZIM/TIFY domain, is responsible for interaction with AtBBD1 (Figure 8E). Therefore these results lead us to conclude that the N-terminal region containing the HCR domain of AtBBD1 interacts with the ZIM/TIFY domain of AtJAZ1 in *Arabidopsis*.

### AtBBD1 Negatively Regulates *AtJMT*

To investigate the *in vivo* function of AtBBD1 in regulating *AtJMT* gene expression, a T-DNA insertion knockout mutant, *atbbd1,* was examined. When treated with MeJA, the *atbbd1* mutant showed no difference from wild type plants (Col-0) in *AtJMT* gene expression (Figure 9A). However, *AtBBD2,* which has 81% amino acid sequence identity to *AtBBD1* (Figure S2C), may have overlapping functions. To test whether these two genes act redundantly, the double knockout mutant, *atbbd1 atbbd2,* was made by crossing the *atbbd1* and *atbbd2* single mutant plants (Figure S2A–B). When the double knockout plants were treated with MeJA, *AtJMT* expression was induced to a higher level and the induction lasted longer than in wild type. In wild type, induction of *AtJMT* transcription by JA was short-lived and transcript levels began to decline after 3 hours of MeJA induction, but in double knockout plants, *AtJMT* transcript levels continued to increase, even 6 hours after MeJA treatment (Figure 9A). The *atbbd1 atbbd2* plants however, showed reduced expression levels of the JA-regulated gene *JR2* in response to MeJA treatment. These results showed that AtBBD1 and AtBBD2 have redundant functions as negative regulators of *AtJMT* gene expression in response to MeJA, but may act as positive regulators of *JR2*.

**Figure 9:** Gene expression pattern in mutants of AtBBD1 and AtBBD2. (A) MeJA response of *AtJMT* in Col-0, *atbbd1,* and *atbbd1 atbbd2* mutants after MeJA treatment. *AtBBD1, AtBBD2* and *JR2* were analyzed by Northern blot, and *AtJMT* was analyzed with RT-PCR. (B) Basal levels of *AtJMT* expression in Col-0, OX-4, and OX-13. (C) MeJA response of *AtJMT* expression between Col-0, OX-4, and OX-13. *AtBBD1* and *JR2* was analyzed by Northern blot and *AtJMT* was analyzed by RT-PCR.

To understand *AtBBD1* function further, *AtBBD1* was overexpressed under the control of the CaMV 35S promoter in transformed lines (Figure S3). Transgenic lines OX4 and OX13, single copy transformants, were selected for further analysis. Consistent with the *atbbd1 atbbd2* mutant phenotype, the basal and JA-induced levels of *AtJMT* expression were lower in OX4 and OX13 compared to wild type (Col-0) (Figure 9B-C). Also, JA-regulated *JR2* gene expression was enhanced in overexpression plants. These results further support the hypothesis that AtBBD1 functions as a repressor of *AtJMT* gene expression *in vivo* by binding to JARE but acts as a positive regulator of *JR2*.

### Chromatin Immunoprecipitation Reveals that AtBBD1 Repression of *AtJMT* is Associated with Histone Deacetylation

To understand the mechanism by which AtBBD1 represses *AtJMT* gene expression, we next examined the level of histone acetylation in the promoter region of *AtJMT*. It has been reported that AtJAZ1 interacts with HDA6 directly and contributes to histone deacetylation [10]. Chromatin immunoprecipitation was carried out with antibodies against modified histones. Fragmented chromatin DNA was incubated with anti-AcH3K14 or anti-AcH4K12 antiserum and isolated DNA was amplified with sets of primers specific to the *AtJMT* promoter region neighboring the JARE (*P_JMT_* ). Upon MeJA treatment, the levels of histone H3 and H4 acetylation in the promoter region of *AtJMT* were enhanced in *atbbd1 atbbd2* mutant plants but reduced in OX-4 compared to wild type plants (Figure 10A). The basal level of histone acetylation in the promoter region of *AtJMT* was also higher in *atbbd1 atbbd2* double knockout plants and lower in OX-4 compared to wild type. qPCR data showed that the histone acetylation level of *AtJMT* was significantly different from wild type, double knockout and OX-4 plants at a confidence level of P<0.05 (Figure 10B). These results showed that AtBBD1 repression of *AtJMT* is associated with histone deacetylation; this deacetylation may occur through the AtBBD1 interaction with AtJAZ1, which was reported to interact with HDA6 [10].

**Figure 10:** Acetylation of chromatin histones associated with *P_JMT_* is enhanced by MeJA. (A) Chromatin immunoprecipitation was carried out with antibodies recognizing acetylated histone H3 (AcH3K14) or H4 (AcH4K12). Precipitated DNA was amplified by primers corresponding to sequences adjacent to the AtBBD1 binding sites in the *AtJMT* promoter (*P_JMT_*). PCR product was analyzed by agarose gel electrophoresis. Actin was used as a control. Input indicates samples before immunoprecipitation. (B) qPCR analysis of ChIP assay with Col-0, *atbbd1 atbbd2*, and OX-4. Open bar is without MeJA treatment and closed bar is with MeJA treatment for 3 hours. Relative fold difference is represented. Statistical significance of the measurements was determined using a t-test (P≤0.05) by comparison with the value for Col-0 (*). Comparison between indicated values is also shown by (**). Data represent the mean values of 3 independent experiments and error bars represent standard deviation.

## Discussion

### Identification of a JARE in the *AtJMT* and *BcNTR1* Promoters

Here we have identified a novel *cis*-element, the JARE, which regulates JA-responsive gene expression and contains a heptanucleotide sequence motif (G/C)TCCTGA. The JARE was identified in two orthologous genes encoding an enzyme involved in JA biosynthesis, −3480 bp upstream of *BcNTR1* and –2290 bp upstream of *AtJMT*, respectively. The same JARE sequence is present in both genes, although at slightly different positions in each promoter. Considering that the two genes are orthologous, encoding the same enzymatic activities in the same plant family, the two loci could have conserved mechanisms of transcriptional regulation in which they share homologous *cis*-acting elements and *trans*-acting factors. The JARE is also found in the promoters of other Arabidopsis JA-responsive genes, including *LOX2, COI1, JAZs (JAZ6, 7,and 8), WRKY70, PDF1.2, VSP1,* and *MYBs (MYB24 and 44)*, and in other plants, including the promoter of the rice JA-responsive gene *OsbHLH148*. Therefore, JA-responsive regulation through the JARE may affect many Arabidopsis genes and may also be conserved beyond the *Brassicaceae*.

The JARE is distinct from other JA-responsive elements previously reported. For example, G-box (CACGTG) and GCC motifs (GCCGCC) are known JA-responsive elements in plants [17], [51]. There are several G-boxes or G-box like elements in the *BcNTR1* and *AtJMT* promoters, but tests of promoter deletions and multimerized JARE constructs showed that these G-box elements are not necessary for the JA response of *AtJMT* and *BcNTR1* expression (Figure 4). Moreover, MYC2 is a TF that interacts with the G-box to regulate JA-responsive genes [15] and *AtJMT* gene expression in response to MeJA treatment was not affected in *myc2* knockout plants (*jin1–7 and jin1–8*) (Figure S4). These results therefore indicate that JA-responsive regulation of *AtJMT* and *BcNTR1* occurs through the JARE and not through G-box elements and suggest that the transcription factors binding to JARE could be different from bHLH transcription factors like MYC2.

The JARE is also distinct from other reported JA-responsive *cis*-elements. For example, the GCC motif was initially defined as an ethylene (ET)-responsive element in EREBPs [52], but it also plays a role in conferring JA- and ET-responsive expression of the *PDF1.2* gene [27]. Also, TGACG sequences were found to be essential for the JA response in promoters of tobacco *nopaline synthase* (*nos*) and barley *lipoxygenase 1* (*LOX1*) genes [53], [54], [30]. JASE1 (CGTCAATGAA) and JASE2 (CATACGTCGTCAA) of *Arabidopsis OPR1* are also reported to be JA-responsive motifs [31]. All of these motifs reported as JA-responsive elements are different from the JARE, which is therefore a novel *cis*-element controlling JA-responsive gene expression.

### AtBBD1 Binds to JARE

To understand the mechanism of *AtJMT* gene expression regulation by the JARE *cis*-acting element, we identified a *trans*-acting factor, AtBBD1, which binds to the JARE. *AtBBD1* is an *Arabidopsis* homologue of *OmBBD1*, which is involved in ABA dependent callose deposition [50]. *AtBBD1* expression was induced by various plant hormones such as MeJA, SA, ABA, and ETP (Figure S5A). The complex regulation of *AtBBD1* indicates that it may act in additional hormonal responses, or in cross-talk among hormonal signaling pathways.

AtBBD1 specifically binds to the JARE sequence, which we defined by mutational analysis as (G/C)TCCTGA, and does not bind to other sequences such as the G-box (Figure 6). Sequence analysis of AtBBD1 did not identify a known DNA binding motif, but Y1H assays revealed that that the AtBBD1 C-terminal domain, containing the UVR domain, binds to JARE. The DNA binding motif of AtBBD1 is also similar to the C-terminal region of DELLA proteins (GAI, and RGA/RGLs) although the DNA binding domain of DELLA proteins has not yet been clearly defined. Consistent with the ability of AtBBD1 to bind DNA, AtBBD1-sGFP fusion proteins were localized in the nuclei of the transformed *Arabidopsis* plants (Figure S5B). Therefore, the characteristics of AtBBD1 are consistent with a role as a nuclear transcription factor.

### AtBBD1 and AtBBD2 Repress *AtJMT* gene Expression

Unlike other JA-dependent transcription factors, which act as transcriptional activators after release from JAZ interaction, AtBBD1 acts to repress expression of the JARE-regulated target gene *AtJMT*. This repression is shown by induction of *AtJMT* expression in mutants lacking both AtBBD1 and its close homologue AtBBD2 (Figure 9 and S6). Y1H assays showed that AtBBD2 binds to JARE (Figure 6) and Y2H assays also showed that, similar to AtBBD1, AtBBD2 interacts with AtJAZ1 and 4 (Figure S7). These results also suggest that AtBBD2 is functionally redundant with AtBBD1. Similar to other JAZ-interacting proteins, the JAZ-AtBBD1 complex could repress *AtJMT* gene expression by recruitment of co-repressors, and by histone deacetylation through interaction between JAZ proteins and HDACs. For example, EIN3/EIL1 directly interact with AtJAZ1 and HDA6 to repress *ERF1* in JA- and ethylene (ET)-responses through histone deacetylation [10].

AtBBD1/2 can also act, directly or indirectly, as positive activator, as shown by increased *AtJR2* expression in the *atbbd1 atbbd2* mutant (Figure 9). Also, Arabidopsis overexpressing *OmBBD1* showed enhanced expression of the JA-related gene *PDF 1.2* and the ABA-related genes *ABA1, RD29*. Considering their narrow spectrum of interaction with JAZs, AtBBD1 and 2 are expected to be involved in a specific subset of JA-related defense signaling, rather than global JA-responses. AtMYC2 interacts with most of the JAZ proteins and is involved in most JA-related phenotypes [21]. By contrast, other TFs involved in specific JA-responses, including TFs such as MYB21/24 and EGL3/GL3/TT8, interact with a small set of JAZ proteins [19], [20]. AtBBD1 might be involved in blocking a MeJA metabolic sink and thus may contribute to increasing the local concentration of JA-Ile, an active form of JA [55]. AtBBD1 could function as a positive regulator responding to JA by post-translational modification or interaction with other proteins [56]. For example, bifunctional TFs, APETALA2 and WUSCHEL, act as activators or repressors on different target genes in plant flower development [57].

Moreover, in addition to, or instead of, acting in initial JA responses, AtBBD1 may act during the recovery after JA induction. Slow induction of *AtBBD1* by JA could reflect its role in the recovery phase. Indeed, the double knockout plant *atbbd1 atbbd2* shows a higher level of *AtJMT* transcript at a later time (Figure 9), indicating a failure of recovery from JA stimulation.

Our results also suggest the existence of a positive regulator or activator responding to JA. For example, induced expression of the multimerized JARE reporter construct (Figure 4) and increased expression of *AtJMT* in the *atbbd1 atbbd2* mutant are consistent with the presence of an activator that also binds the JARE. Although we did not find such an activator by Y1H hybrid screening, it is possible that the specific activator could compete with AtBBD1 for binding to the JARE. The postulated positive regulator may also be subject to JAZ-dependent regulation, as *AtJMT* expression is still strongly induced by JA in the *atbbd1 atbbd2* mutant plants.

Regulation by competing positive and negative transcription factors has substantial precedent. In plants, a family of transcription factors, such as the auxin-responsive element binding factors (ARFs) or ET-responsive element binding factors (ERFs), can share the same DNA binding domain and the same *cis*-element, but many of the members have opposite functions in target gene regulation [58], [59], [60]. For example, ERFs bind to the same *cis*-element (GCC-box) but regulate target gene expression in the opposite manner. ERF1, 2, and 5 function as activators and ERF3, 4, and 7–12 function as repressors [58], [61]. Their repression activity is conferred by the EAR motif in ERF3 and 4 [61], [62]. The EAR motif interacts with the corepressor TPL. ERF-TPL complexes repress target genes by modification of chromatin structure through histone deacetylase [39]. In the case of ARF family TFs, ARF5–8 and 19 activate target gene expression and the others repress target gene expression although they bind to the same auxin-responsive *cis*-element [59]. ARFs require the association with Aux/IAA repressors for an auxin response [59], [60]. Many Aux/IAA proteins are degraded by the SCF^TIR1^ complex in an auxin-dependent manner [63]. These examples are reminiscent of the mechanism of JA signal transduction through JARE. Therefore, it is possible that AtBBD1 could bind to the JARE as a repressor and that other TFs with a similar DNA binding domain could compete with AtBBD1 and act as activators.

In conclusion, the mechanism of AtBBD1 negative regulation of *AtJMT* could be postulated to function as follows (Figure 11); AtBBD1 recognizes the JARE in the *AtJMT* promoter and interacts with AtJAZs. When the JA signal is absent, the AtBBD1-AtJAZ complex recruits co-repressors or HDACs. Putative activator also competes with AtBBD1 for binding to the JARE; in the absence of JA, this activator may be bound by JAZs. When the JA signal comes in, JAZs are degraded by the 26S proteasome pathway through SCF^COI^, and AtBBD1 is then released from JAZs. At the same time, the activator is also released from JAZs and activates *AtJMT*. The *AtJMT* expression level is regulated by the balance between activator and AtBBD1. In knockout plants, the activator occupies the JARE and *AtJMT* gene expression is activated to higher levels than wild type because the AtBBD1 repressor is absent. In AtBBD1-overexpressing plants, AtBBD1 occupies the JARE dominantly over the activator and *AtJMT* gene expression is repressed more than in wild type. Identification of putative activator protein interacting with JARE would fill out the model more precisely.

**Figure 11:** Proposed model for transcription repression by AtBBD1. In the absence of signal, AtBBD1 represses *AtJMT* gene expression by recruiting corepressor or HDAc through AtJAZ. In the presence of signal, JA-Ile is released and the SCF^COI1^ complex degrades JAZ proteins. A putative activator (+) that binds to the JARE competes with AtBBD1 (repressor). In knockout plants, the putative activator dominantly occupies the JARE and *AtJMT* gene expression is activated higher than wild type. In the AtBBD1-overexpressing plant, AtBBD1(repressor) competes with the putative activator and dominantly occupies the JARE; therefore, *AtJMT* gene expression is repressed more than in wild type. Size of each circle represents relative abundance.

## Supporting Information

Figure S1 **DNA binding ability of AtBBD1.**
(TIF)

Figure S2 **Analysis of** ***atbbd1*** **and** ***atbbd1 atbbd2*** **knockout lines.**
(TIF)

Figure S3 **Analyses of transgenic** ***Arabidopsis*** **overexpressing** ***AtBBD1.***
(TIF)

Figure S4 ***AtJMT*** **expression pattern in** ***myc2*** **mutants.**
(TIF)

Figure S5 **Expression pattern and localization of AtBBD1.**
(TIF)

Figure S6 **Gene expression pattern in** ***atbbd2*** **mutant.**
(TIF)

Figure S7 **Interaction of AtBBD2 with AtJAZ1 and AtJAZ4 in yeast.**
(TIF)

Table S1 **List of constructs and primer sequences used in this study.**
(PDF)

Procedure S1 (PDF)
